RETRACTED

# A Novel Diabetes Healthcare Disease Prediction Framework Using Machine Learning Techniques

**DOI:** 10.1155/2022/1684017

**Published:** 2022-01-11

**Authors:** Raja Krishnamoorthi, Shubham Joshi, Hatim Z. Almarzouki, Piyush Kumar Shukla, Ali Rizwan, C. Kalpana, Basant Tiwari

**Affiliations:** ^1^Department of ECE, Vignan's Institute of Management and Technology for Women, Kondapur (V), Ghatkesar (M), Medchal-Malkajgiri (D), Padamatisaiguda, Telangana 501301, India; ^2^Computer Engineering, SVKM'S NMIMS, MPSTME Shirpur Campus, Savalade, India; ^3^Department of Radiology, Faculty of Medicine, King Abdulaziz University Hospital, Jeddah, Saudi Arabia; ^4^Computer Science & Engineering Department, University Institute of Technology, Rajiv Gandhi Proudyogiki Vishwavidyalaya (Technological University of Madhya Pradesh), Bhopal 462033, India; ^5^Department of Industrial Engineering, Faculty of Engineering, King Abdulaziz University, Jeddah 21589, Saudi Arabia; ^6^Dept. of CSE SST College of Art and Commerce, Ulhasnagar, India; ^7^Ethiopia Hawassa University, Awasa, Ethiopia

## Abstract

Diabetes is a chronic disease that continues to be a significant and global concern since it affects the entire population's health. It is a metabolic disorder that leads to high blood sugar levels and many other problems such as stroke, kidney failure, and heart and nerve problems. Several researchers have attempted to construct an accurate diabetes prediction model over the years. However, this subject still faces significant open research issues due to a lack of appropriate data sets and prediction approaches, which pushes researchers to use big data analytics and machine learning (ML)-based methods. Applying four different machine learning methods, the research tries to overcome the problems and investigate healthcare predictive analytics. The study's primary goal was to see how big data analytics and machine learning-based techniques may be used in diabetes. The examination of the results shows that the suggested ML-based framework may achieve a score of 86. Health experts and other stakeholders are working to develop categorization models that will aid in the prediction of diabetes and the formulation of preventative initiatives. The authors perform a review of the literature on machine models and suggest an intelligent framework for diabetes prediction based on their findings. Machine learning models are critically examined, and an intelligent machine learning-based architecture for diabetes prediction is proposed and evaluated by the authors. In this study, the authors utilize our framework to develop and assess decision tree (DT)-based random forest (RF) and support vector machine (SVM) learning models for diabetes prediction, which are the most widely used techniques in the literature at the time of writing. It is proposed in this study that a unique intelligent diabetes mellitus prediction framework (IDMPF) is developed using machine learning. According to the framework, it was developed after conducting a rigorous review of existing prediction models in the literature and examining their applicability to diabetes. Using the framework, the authors describe the training procedures, model assessment strategies, and issues associated with diabetes prediction, as well as solutions they provide. The findings of this study may be utilized by health professionals, stakeholders, students, and researchers who are involved in diabetes prediction research and development. The proposed work gives 83% accuracy with the minimum error rate.

RETRACTED

## 1. Introduction

Of late, diabetes is one of the leading reasons for death in developing countries. To find the solution for the crucial disease, the government and individuals are investing money in research studies. Diabetes is a disease in which blood sugar levels continue to rise due to a lack of insulin, which affects blood sugar metabolism. Diabetic patients cannot effectively convert consumed carbohydrates into glucose sugar that produces energy for day-to-day activities. This leads to a gradual increase in sugar in the bloodstream. Therefore, glucose remains in the bloodstream and will not reach all body cells [1].

Hence, it remains a challenge to predict as it involves different parameters. Prediction and detection of disease are made by adopting many predictive, quantitative, and statistical models. In recent times, diabetes becomes one of the leading causes of death in developing countries. Mainstream research has been funded to enhance analysis in the following fields and is driven by the emotive to find quick solutions. Diabetes is one of the most prevalent diseases that develops as a result of a high amount of blood glucose or blood sugar in the bloodstream. The glucose in the blood is the most important energy source for the human body, providing it with the energy it needs to complete the full task. This energy is derived through insulin, which is produced with the assistance of the pancreas, which obtains energy from the consumption of food. As soon as a patient is diagnosed with diabetes, the glucose is unable to reach any cells in the body, which has an impact on the whole body's functioning. According to the findings of the study, 30.2 million individuals in the United States are suffering from diabetes. This diabetes contributes to the development of further diseases such as heart disease, stroke, and other health issues. In this section, we will cover diabetic [2] difficulties that may affect someone as early as infancy and lead them to gain weight as a result of cells that are no longer functioning properly.

RETRACTED

Healthcare industries have a massive number of databases consisting of different types of data such as structured, semi-structured, or unstructured. According to the healthcare sector, ER data sets are too huge. Big data analytics can process and analyze the large volume of data sets and discover hidden patterns and information and complex to be processed by traditional techniques. The application of predictive analytics in the healthcare sector has received a great amount of interest in the research community [3].

Type 1 diabetes is the most common type of diabetes, and it occurs when the human body does not produce enough insulin. The low insulin production as a result of both immune system attack and loss of pancreatic function is a prevalent occurrence in the diabetic population. This type of diabetes has been seen in both children and adults, according to the research. They must consume an adequate amount of insulin to secure their continued existence on this planet. The most significant risk factors for type 1 diabetes include family history, pancreatic illness, and pancreatic infection. Type 2 diabetes is the following stage, and it occurs when the body's insulin is not appropriately used. This type of diabetes may afflict persons of any age, although it is most typically seen in adults in their middle years. According to the National Institute of Diabetes Digestive Kidney Center, type 2 diabetes is associated with the development of an obesity problem in the population. Fatigue and insulin resistance are associated with type 2, as are poor glucose tolerance and gestational diabetes. Other type 2 risks include ethnic origin, sedentary lifestyle, age, insulin resistance, and PCOS. Along with diabetes, prediabetes is a condition that affects humans when their blood sugar level falls between 100 and 124 milligrams per deciliter (mg/dL). When it comes to glucose levels, prediabetes is characterized as having a higher level than other types of diabetes but not as high as other types of diabetes. Indeed, insulin is an insulin-secreting pancreatic hormone that plays an important role in allowing blood sugar to be utilized as energy in cells. When a person has prediabetes, the cells of the body do not normally respond to insulin in the same way. The pancreas produces more insulin in an effort to induce cells to respond on a consistent basis. The pancreas will eventually be unable to keep up, and blood sugar levels will rise, paving the path for the development of prediabetes and, eventually, type 2 diabetes.

RETRACTED

The latest development of ML has increased the capacity of the computer system to recognize and label images, predict diseases, and improve decision-making by analyzing the data. The objective of ML applications is to train the computer system to perform better than a human being. The supervised learning algorithm is used for training the model, and evaluation is done using testing data [4].

The method of detecting diabetic illness is shown in the diagram above, and it contains numerous processes such as diabetes data collecting, noise data removal, feature extraction, selection, and disease classification, among other things. Optimized techniques are used to predict the diabetes sickness in line with the general stages, and there have been no complications.

The data play a very important role in machine learning, and it is really important. In practically every industry, including medical, education, and transportation, there is a wealth of information accessible. These data, in turn, give knowledge that is extremely helpful in assisting individuals in making more informed decisions. The usage of data in the retail industry is used to forecast the purchasing behaviors of clients.

Using knowledge gleaned from retail market data, it is feasible to increase the number of items being produced. It is possible to evaluate transportation data in order to simplify the transportation process without causing any disruptions. In a similar vein, data available to the medical profession may be evaluated to predict diseases in advance, allowing for a greater number of lives to be spared. In hospitals, there is a huge quantity of information available on the patients. When these data are correctly retrieved, they may provide even more insights that can be used to anticipate illnesses months or even years in advance. In machine learning, models are formed based on the data that have been gathered and processed.

According to the participants in the conference, data collecting is critical when assessing the diabetic illness. As a result, the Pima Indian Diabetes Database data set is used in this study to investigate the condition of diabetes.

Diabetic illness is the most prevalent disease that affects humans. It is caused by an inadequate synthesis of insulin and excessive blood sugar levels in the blood. Before doing a clinical examination, it is necessary to look for many signs and symptoms of diabetes. Although the newly discovered symptoms are basic to detect in a handbook, the accuracy of diabetes prediction continues to be a serious challenge. Although newly discovered symptoms are easy to access in a handbook, the accuracy of diabetes prediction continues to be a significant challenge. There are several researchers that are devoted to this topic, with the goal of accurately diagnosing diabetic condition via the collection of large amounts of data. The standard stages for recognizing diabetic illness make use of the smallest amount of processes possible, but they fall short of achieving the highest possible detection accuracy.

RETRACTED

To manage the challenges stated above, the different writers' opinions, templates, and paper works are taken into consideration in order to get an understanding of the diabetic illness detection process.

Improved approaches are developed to construct a hybrid early diabetic illness prediction system based on the information gathered from the various authors' works. The newly developed algorithm takes advantage of publicly accessible diabetic data to anticipate the changes accurately. As a result, the system successfully detects the diabetic illness by reducing the number of false positives.

Different ML algorithms can be applied to the different structures of data. This study examines predictive analysis in the healthcare sector. ML algorithms are applied to healthcare data sets for analysis. This experiment is centered on gestational diabetes in the study. KNN, SVM, logistic regression, and random forest ML techniques are performed on the Pima Indian Diabetes Database (PIDD) data set to investigate the prediction of diabetes. The test is conducted by taking various parameters such as glucose, blood pressure, and BMI [5] to achieve precision. The remaining work is bestowed as follows.  Section 3 describes diabetes prediction's related work.  Section 4 discusses the overview of classification algorithms. Experimental results are presented in Section 5. Finally, a brief paper of conclusion is discussed in Section 6.

## 2. Related Work

This section discusses the different strategies and procedures that may be used to anticipate the development of diabetes. An effective diabetes analysis model was developed using K-means clustering with support vector machine (SVM) training data to achieve success [6]. During the information investigation process, diabetes information is acquired from the University of California, Irvine Pima Indians Diabetes data set, and hidden instances, and missing characteristics are evacuated using the commotion expulsion technique to the data set. In addition, the commotion-free information is created using a K-means bunching procedure that selects the best features, and the *t*-test is carried out using the assist vector machine to reduce the amount of noise. The efficiency of the framework is being evaluated based on the results of exploratory studies.

RETRACTED

With the use of the binary PSO approach, many medical disorders have been investigated utilizing various data sets such as the PIMA Indian Diabetes Database data set, the heart database, the dermatology data set, and the Wisconsin breast cancer data set. The newly presented optimized approach checks four data sets for relevance, and the relevant features are picked based on the location and velocity value of the feature positions. The chosen characteristics aid in the prediction of the associated medical illness without adding any further complication. The system's effectiveness is then evaluated in terms of accuracy, information gain, and F score value, all of which are greater when compared to the typical genetic feature selection method, which is next evaluated [7].

An intelligent strategy for enhancing the accuracy of diabetes diagnosis was described with the use of an adaptive neuro-fuzzy inference system (ANFIS) and principal component analysis (PCA). The PCA algorithm is used to reduce the amount of characteristics included in the diabetes data set, to be more particular. For the early diagnosis of diabetes, the ANFIS classification model is essential [8]. The ANFIS classification model is developed on the basis of reduced characteristics [9].

Diabetes data have been examined using a variety of data mining approaches, including SVM, integrated learning model, and the decision tree approach [10]. Initially, the data were collected from individuals who were examined using the SMOTE algorithm, which is one of the most effective feature selection algorithms, in conjunction with an imbalanced approach, which selects features such as BMI, glucose level, and age while not eliminating other important features such as smoking status. When the chosen features are processed, they are examined by the data mining classifier described above, which distinguishes between normal and abnormal characteristics without causing any failures.

The accuracy and precision of the SMOTE-based diabetes identification system are greater than those of classic support vector classifiers, with a ROC value of 0.9817% and 94.65% accuracy rate, respectively. It is said in the discourse that the opinions of various creators are pooled in individual management initiatives to get knowledge and ideas about the diabetic condition forecasting method.

Several researchers, including [11], have expressed concern that most present diagnostic models are constructed to have a knowledge base collecting hospital data and symptoms associated with a certain ailment. The correctness of the knowledge base has a significant impact on the performance of the prediction system. To address this issue, a rough set-based prediction system was developed and put into operation. The suggested approach makes use of the symptoms provided by 19 individuals as input to determine the type of diabetes that they have. It has been shown that the outcomes of the rough set-based prediction models are much better than those of the current rule-based prediction models.

RETRACTED

It is required to modify the settings of learning algorithms in order to improve the output of difficult optimization issues [12]. In addition, it was revealed that the optimization method is becoming a popular alternative for solving complicated issues that are very difficult to address using conventional techniques. Fuzzy logic with PSO, GSA, and ACO may be used to tackle challenges that are currently encountered with machine learning approaches.

Fuzzy logic and PSO were used in the prediction of cardiovascular disease, and the results were published in science. The developed approach makes use of decision trees to choose the most essential attributes from the UCI data set that will be most helpful in forecasting the disease's occurrence. The conclusion of the decision tree is turned into fuzzy rules, which are then optimized using the PSO algorithm [13].

With the use of artificial neural network colony optimization and fuzzy logic, researchers have developed a novel categorization strategy that may assist clinicians in improving the diagnosis of diabetic condition [14].

It was necessary to increase the performance efficiency of machine learning methods in two stages [15]. It is necessary to choose the most relevant characteristics in the first stage, which is accomplished using a correlation-based feature selection method. The random forest technique is used to categorize heart disease and diabetic illness in the second stage. Following analysis of results, it was discovered that the suggested random forest technique considerably improves the prediction efficiency of heart disease and diabetic illness.

The different side effects produced by diabetic illness were discussed, as well as the need of diagnosing diabetic disease at an early stage in the disease's progression. Nevertheless, it has been suggested that detecting diabetes at an early stage may aid diabetic patients in diminishing their chance of developing other illnesses such as heart disease, neuropathy, or retinopathy in the future. A multilayer neural network is utilized to improve the effectiveness of a diabetes prediction system, according to the researchers.

The complexities of diabetic illness were discussed, as well as the need and relevance of intelligent systems in better anticipating the diabetes disease's progression. To improve the accuracy of diabetes prediction, LDA is used to choose more relevant aspects that are closely associated with the condition of diabetes. The adaptive neuro-fuzzy interference system is then used to classify the data based on the characteristics that have been chosen before. It has also been claimed that the proposed method might be utilized by physicians as a cost-effective tool to help them make more accurate judgments.

RETRACTED

Zou et al. [16] postulated about prognostic analytics in health care and used six ML techniques on the data set. The evaluation was done and compared with different ML models to predict diabetes. The performance of SVM and KNN had high accuracy for the PIDD data set. However, the work did not consider hyper-parameter tuning models for obtaining high accuracy.

Wang et al. [17] discussed the structured framework for predicting diabetes using the ML algorithms. However, in the existing system, the classification and accuracy were not so high. They proposed a pipeline model for diabetes prediction and to increase the classification accuracy. Haseen et al. [18] explained about classifying the diabetes mellitus risk. Four ML algorithms decision tree, ANN, logistic regression, and naive Bayes were examined. Later, the Bugging and Boosting techniques were adopted to enhance the robustness of the models. After evaluation, the random forest was considered as best for disease.

### 2.1. Risk Classification

Srinivasan et al. discussed the complication of diabetes if it is untreated. Investigating diabetes is a tedious diagnosing process. ML approaches were framed to solve this problem. Three ML techniques such as decision tree, SVM, and naive Bayes are used on the PIMA data set. 76.30% of accuracy was achieved while comparing with another algorithm. Finally, the proposed framework of NN unfolds split prediction to achieve 84.52% of accuracy.

## 3. Methodology

The proposed framework is divided into different phases. The flow diagram is illustrated in Figure 1. Python Jupyter Note was used for the entire implementation. Different packages such as NumPy, pandas, scikit, and Matplotlib have been used in analyzing the data. The task performed in each phase and the relevant functions explored from Python tool kits are described below.

### 3.1. Data Set (PIDD)

Pima Indian Diabetes Database is a familiar and commonly used data set for the prediction of diabetes. This data set consists of 768 rows and 9 columns. The attributes included in the column are glucose, pregnancies, skin thickness, blood pressure, BMI, insulin, age, and outcomes. The outcome variable predicts whether the patient is diabetic [19] positive or diabetic-negative. Pandas function is utilized to read CSV.file where the data set file is in excel format.

RETRACTED

### 3.2. Data Visualization

Data visualization helps to understand the data better by putting it in a visual form. In this phase, data are represented in the form of bar chart. The analysis reveals the percentage of people affected by diabetes diseases. It also displays the information of the data set such as age, blood pressure, pregnancies, and glucose. Apart from that, it predicts how many people are affected by diabetes from 768. For displaying output, the graphical representation functions such as plot axis, pyplot, and several others have been used.

### 3.3. Preprocessing

This section includes the removal of outliers and standardizing the data. The processed data have been used for creating a model. The data should be preprocessed and arranged properly before applying classifiers to the data index. These data should be handled carefully before connecting.

In this phase, inconsistent data are handled and removed to obtain more precise and accurate results. This data set contains missing values. Few selected attributes such as blood pressure, skin thickness, glucose level, and BMI are assigned with missing values because these parameters cannot have null values. Then, we normalized all values by scaling the data set.

### 3.4. Machine Learning Classification Algorithms

Subsequently, after preprocessing the data ML classifiers are applied using the scikit-learn Python Toolkit. Scikit is a simple tool kit used to process and analyze the data [20]. These tool kits are used in most of the work. Foremost using a function like the model selection train test split, the data set is divided into the training and testing data sets. Due to the limited data set source, about 90%, of the data set, is used for training purposes and the remaining 10% is used for testing by selecting the data randomly. Then, different classifiers such as ML algorithms [21] are applied to diagnose diabetes. ML classifiers are adapted because of their simplicity and popularity. Since this work focuses on hyper-parameter tuning, it will be explained in the succeeding section.

### 3.5. Hyper-Parameter Tuning

Hyper-parameter tuning is used to evaluate the ML models. The process of choosing a set of optimal hyper-parameter is known as hyper-parameter tuning [22]. The value of the hyper-parameter's model is fixed before starting the ML task. Hyper-parameter tuning plays a significant role in ML techniques. The model parameters are secured from the data. For getting the best fit, hyper-parameter tuning is performed. Selecting the best hyper-parameter is a complex problem, so grid search and random search algorithms are used. This technique is adapted to increase the accuracy of the ML classifier [23].

RETRACTED

### 3.6. Comparison

In this section, the ML classification algorithm is compared based on accuracy. After the evaluation process, one of the best ML classifiers is identified and hyper-parameter tuning has been applied to produce the best result.

### 3.7. Performance Evaluation

In the last section, the performance of the logistic regression classifier will be assessed by adapting execution measurements such as ROC, precision, and test score. The generated result is then compared with the relevant work for performing result analysis [24].

## 4. Machine Learning Classification Models

### 4.1. Logistic Regression (LR)

LR models have been acquired from the statistics branch. This algorithm has adapted for binary classification problem statements. The main aim of LR is to discover the value of coefficients. The LR converts the value to 0-1. LR model selects the probability of the given data instance of the class to predict as 0 or 1. This technique can be applied for problems when we emerge with multiple reasons for predicting.

The LR standard function is defined as follows:

(1) $$\begin{array}{c} h\theta \left(X\right)=\frac{1}{1+e^{-\left(\beta_{0}+\beta_{1}X\right)}}. \end{array}$$

Equation (1) represents the logistic decision of the predicted data. X is the data label where the constants are represented in *β*_1_ and *β*_0_.

### 4.2. K-Nearest Neighbor (KNN)

KNN is one of the ML supervised learning techniques [25]. It is mostly applied in classification problems. KNN is used to classify objects depending on the closest measure/distance, i.e., the distance between the object and all objects of training data. Based on K-neighbors, the item is classified. Positive integer K is defined before executing the algorithm. Very often Euclidean distance is used to calculate the different measures of the objects [26]. The calculation of the Euclidean distance equation is given below:

(2) $$\begin{array}{c} \text{Euclidean}\sqrt{{\sum_{i=1}^{k}{\left(x_{i}-y_{i}\right)}^{2}}^{}}, \end{array}$$

(3) $$\begin{array}{c} {\text{Manhattan}\sum_{i=1}^{k}\left|x_{i}-y_{i}\right|}^{}. \end{array}$$

From equations (2) and (3), Euclidean and the Manhattan of the KNN classifier are found with the x and y data up to i variables.

### 4.3. Support Vector Machine (SVM)

SVM algorithm is a supervised ML technique [24]. This model is desirable for a small data set that has few outliers. The key is to identify the hyperplane to divide the data points. The identified hyperplane will separate two spaces into various domains. Such domain will consist of similar types of data.

(4) $$\begin{array}{c} ||x||=\sqrt{x_{1}^{2}+x_{2}^{2}+\cdots +x_{n}^{2}}. \end{array}$$

Equation (4) represents the decision state of the support vector machine. A hyperplane separates the space into two sectors. The hyperplane is a binary classifier, and it is applied to linear classification [27]. The subspace of a single dimension will be less than its circumstances.  Figure 2 demonstrates SVM hyperplane classification.

RETRACTED

### 4.4. Random Forest

Random forest is an ML algorithm, and it belongs to the supervised learning model. RF classifier consists of several decision trees of the different subjects from the given data set. To improve the predictive accuracy [28], it takes the average from the subset from each tree. RF takes majority vote prediction from all the trees and finally predicts the output rather than relying on one decision tree. Every node decision tree executes a question concerning the data.

### 4.5. Proposed Framework Logistic Regression

Hyper-parameter tuning was proposed. Hyper-parameter tuning ML models are parameterized, and based on the problem statement, the behavior can be tuned. Models can have various parameters/attributes. Identifying the prime fusion of attributes can be considered a search problem. LR tuning used two strategies: grid search and random search. The random search identifies sample distribution for all parameters and defines the number of iterations required for searching the optimal model. The values of the hyper-parameter are selected by sample distributions. In our work, we applied a grid search.

(5) $$\begin{array}{c} \begin{array}{c} \underset{w,b}{\text{min}}\left\{-\frac{1}{n}\overset{n}{\underset{i=1}{\sum }}\text{Pr}\left(y_{i}=1|x_{i};w,b\right)+ℛ\left(w\right)\right\}\\ \text{R}\left(w\right)=\lambda \left\{\alpha \overset{p}{\underset{i=1}{\sum }}\left|w_{i}\right|+\frac{\left(1-\alpha \right)}{2}|w{|}^{T}L|w|\right\} \end{array}. \end{array}$$

Equation (5) represents the grid search algorithm. In grid search, the ML model R takes hyper-parameters x1, x2, and x3. We have to define the values of x1, x2, and x3 hyper-parameters. The grid technique will develop many R versions with the probable hyper-parameter value combination (x1, x2, x3), which was determined in the first place. This type of hyper-parameters value can be tuned as grid.

During grid search, it isolates all parameters and looks for the best probable value while keeping the rest of the parameter constant. It resulted from the model score being less effective. When compared to random search, it showed more improved exploratory power. Because of this power for the critical range, it was able to find the optimal value (hyper-parameter). In this research work, we have applied grid search to increase the effectiveness and efficiency [29] of the LR classifier and to improve the accuracy of the prediction model.

RETRACTED

### 4.6. Result and Evaluation

PIDD data set consists of 768 patients of which 268 patients were affected with diabetes and 500 patients are nondiabetic.  Figure 3 represents the bar chart comparison of proposed technique.

After completing data processing, the training data set is divided. Four ML classifier algorithms were applied. Hyper-parameter tuning and cross-validation were performed to get optimum results for the given data set. As explained previously for ML algorithms, KNN, LR, SVM, and RF were applied. The hyper-parameter tuning and the results obtained from all models are described below. The performance of ML algorithms is examined by different evaluation metrics such as B1 score, recall, precision, and accuracy [30]. The equation is given below:

(6) $$\begin{array}{c} \text{sensitivity}=\frac{TP}{TP+FN}\times 100,\\ \text{specificity}=\frac{TN}{TN+FP}\times 100,\\ \text{accuracy}=\frac{TP+TN}{TP+FP+TN+FN},\\ \text{PPV}=\frac{TP}{TP+FP}. \end{array}$$

- True negative (TN): when it is (F), the samples can be classified or false (F)
- False positive (FP): when it is (F), the samples can be classified as (T)
- False negative (FN): when it is (T), the sampled can be classified as (F)

### 4.7. Analysis of Results Using Different ML Techniques

In this work, four classifier models such as LR, RF, SVM, and KNN were built. Before training the data, the set outlier was eradicated. ML algorithm comparison is indicated in the bar chart.  Figure 3 indicates that RF and SVM have a high accuracy of 83%. After applying hyper-parameter to LR, we were able to improve the accuracy level of prediction by 3% [31].  Figure 4 illustrates the correlation of the confusion matrix. It determines the output result for filling missing values and outlier rejection values simultaneously. The correlation attribute with the target variable depicts that the correlation coefficient has improved remarkably, summarizing statistical data using a box plot. The given data summarize the five numbers such as maximum, minimum, first quartile, median, and third quartile. The presence of null value in the BMI and blood sugar needs to be eradicated in the data preprocessing section. By analyzing BMI and pregnancies (as per Figure 5), we find the existence of a strong positive connection between BMI and the number of pregnancies [32]. A person who was diagnosed diabetic-positive had a high BMI when compared with a nondiabetic person. There is not much difference among the medians. Generally, women who had more pregnancies had high BMI [33]. The relationship between pedigree function and clinical test reports shows that people having high pedigree function are tested positive and the person tested negative had low pedigree function.

RETRACTED

Since the person who tested positive are having a high median and outliers, the pedigree function helps to estimate the diabetic test results accurately. It shows that diabetes is a hereditary disease. We conclude that the genetic component significantly contributes more to the evolution of diabetes in the PIMA Indians Diabetes data set.  Figure 6 illustrates that the significant difference in the average number of pregnancies is high (4.9) in diabetic women while compared to that (3.3) in nondiabetic women.

Figure 7 represents that the women who are weighed normal have 9 times the risk of diagnosing diabetes when compared to the overweighed women. BMI is considered high for the interquartile range of the women who had tested positive.

Women who are above 31 years of age group are at high risk of diagnosing diabetes when compared to the young age.

Figure 8 provides the confusion matrix of the proposed work. Each data layer's number points are classified by the diagonal elements of the matrix. The accuracy can be calculated by the sum of the components on the diagonal divided by the sum elements of the entire matrix. A model can be considered as a good model only if it has a confusion matrix big value on the main diagonal and a small value on the rest of the matrix.

The receiver operating characteristic (ROC) plot is used to evaluate the performance of the algorithm. ROC has been applied successfully in healthcare prognosis and diagnosis. A system/model can be considered a good method if the reference point focuses on the upper defer corner of the ROC chart [34]. The reference points will help us understand the highly sensitive and have fewer FP reference values. The area below ROC is the best way to normalize (known as AUC—area under the curve). If the method has an AUC above 0.5, then we can consider it as a good test method.  Figure 9 represents the ROC value of LR. 86% attained high value when compared to others [35]. We can conclude that RF is suitable for predicting disease with high accuracy.

Figure 9 represents the ROC of the proposed logistic regression. ROC of the proposed work increases during the training phase. Some of the training data may mismatch during the training phase, which results in error rate.

## 5. Summary and Conclusion

ML technique is considered valuable in diagnosing the disease. Early diagnosis advantages the patients with early medical attention. In this study, few existing ML classification models for the prediction of diabetic patients have been discussed based on the accuracy. An expression of accuracy on the classification problem has been identified. ML technique was enforced on the PIDD data set. It was trained and confirmed on the test data set and verified. The results of our implementation method show how the LR performed better than other Ml algorithms. The results show that glucose and BMI strongly correlate with diabetes using association rule mining. It has been found that the ROC value of LR is 86%. The drawback of the study is that we have selected a structured data set, and the unstructured data will be considered for the future. The models can be implemented or suggested to other healthcare domains for the prediction of cancer, Parkinson's disease, heart disease, and COVID-19. The further scope of the research is to consider other attributes such as family history of diabetes, smoking habit, drinking habit, and physical inactivity for the prediction of diabetes.

RETRACTED

## 6. Future Work

Our plans for future work include developing an Android application for the suggested hypothetical diabetes monitoring system, including the proposed categorization and prediction algorithms, and deploying it. Genetic algorithms, in conjunction with the suggested prediction mechanism, may be investigated for improved monitoring.

## Figures and Tables

**Figure 1:** Framework of ML techniques.

**Figure 2:** SVM classification. (a) SVM hyperplane classification. (b) SVM identification of the right hyperplane. (c) Identification of the right hyperplane. (d) SVM classification of two classes.

**Figure 3:** Representation of the bar chart of this data set.

**Figure 4:** Analysis of correlation between variables.

**Figure 5:** Analysis between BMI vs pregnancy vs diabetes variables.

**Figure 6:** Existing association between the test result and the pedigree function.

**Figure 7:** BMI had a close association with the occurrence of diabetes.

**Figure 8:** Confusion matrix of ML algorithms.

**Figure 9:** ROC of logistic regression.

## Data Availability

The data that support the findings of this study are available on request from the corresponding author.
